The article "By downregulating TIAM1 expression, microRNA-329 suppresses gastric cancer invasion and growth" was retracted in 2026. Reasons: plagiarized images; duplicated images; overlap with other authors' work; unreliable results or conclusions.

# By downregulating TIAM1 expression, microRNA-329 suppresses gastric cancer invasion and growth

**DOI:** 10.18632/oncotarget.2755

**Published:** 2015-02-19

**Authors:** Zheng Li, Xin Yu, Yang Wang, Jianxiong Shen, William Ka Kei Wu, Jinqian Liang, Fan Feng

**Affiliations:** ^1^ Department of Orthopaedic Surgery, Peking Union Medical College Hospital, Chinese Academy of Medical Sciences and Peking Union Medical College, Beijing, China; ^2^ Department of Abdominal Surgery, Cancer Institute and Cancer Hospital, Peking Union Medical College and Chinese Academy of Medical Sciences, Beijing, China; ^3^ Department of Anaesthesia and Intensive Care, The Chinese University of Hong Kong, Hong Kong, China

**Keywords:** Gastric cancer, MicroRNAs, miR-329, TIAM1

## Abstract

Gastric cancer (GC) is one of the most common malignant tumors worldwide. Emerging evidence has shown that abnormal microRNAs (miRNAs) expression is involved in tumorigenesis. MiR-329 was previously reported to act as a tumor suppressor or oncogene in some types of cancer. However, its function in gastric cancer (GC) is unclear. Here, we found that miR-329 was down-regulated in GC compared with adjacent controls. Enforced expression of miR-329 inhibited proliferation, migration and invasion of gastric cancer cells *in vitro*. We identified T lymphoma invasion and metastasis 1 (TIAM1) gene as potential target of miR-329. MiR-329 levels inversely correlated with TIAM1 expression in GC. Importantly, TIAM1 rescued the miR-329-mediated inhibition of cell invasion and proliferation. Finally, reintroduction of miR-329 significantly inhibited tumor formation of GC in the xenograft mice. Our findings suggest that miR-329 is a tumor suppressor and potential therapeutic target of GC

## INTRODUCTION

Gastric cancer (GC) is the fourth most commonly diagnosed cancer and the second leading cause of cancer deaths worldwide [1, 2]. Despite the significant achievements in the treatment of early GC, the long-term survival rate for advanced GC is still quite low [3, 4]. Metastasis leads to most of the mortalities and has a critical role in the poor prognosis [5, 6]. However, the underlying molecular mechanisms underlying the invasion and metastasis of advanced GC are still poorly understood [7]. Hence, it is urgent to identify important molecules in GC metastasis and progression, which may be used to develop novel avenues for drugs targeting these markers.

The microRNAs (miRNAs) are an abundant class of small non-coding RNAs, which are single stranded and consist of 19–25 nucleotides [8, 9]. MiRNAs can suppress gene expression at the post-transcriptional level by blocking mRNA translation or degrading target mRNAs through binding to the 3′ untranslated regions (UTR) of target mRNA [10–12]. Mounting evidence has shown that miRNAs are abnormally expressed in various cancers and deregulated miRNAs are associated with tumor initiation, promotion, and progressions [13–17]. In particular, miRNAs can function as tumor suppressors or oncogenes that regulate various cellular processes of tumor cells, including differentiation, progression, apoptosis, and proliferation [5, 18–20].

The article "By downregulating TIAM1 expression, microRNA-329 suppresses gastric cancer invasion and growth" was retracted in 2026. Reasons: plagiarized images; duplicated images; overlap with other authors' work; unreliable results or conclusions.

MiR-329, which is located on 14q32.31, is reported to be downregulated in several cancers, including neuroblastoma and glioma multiforme [21–23]. MiR-329 can suppress neuroblastoma cell growth and motility partially by targeting KDM1A [22]. Moreover, miR-329 may inhibit cell proliferation in human glioma cells through regulating E2F1-mediated suppression of Akt pathway [23]. However, the function and molecular mechanism of miR-329 in human GC are elusive. In this study, we aimed to determine the expression and function of miR-329 in GC and investigate the molecular mechanism of miR-329 in GC cells.

## RESULTS

### miR-329 was down-regulated in GC

As shown in Figure 1A, the expression of miR-329 was significantly down-regulated in four cell lines (MGC-803, SGC-7901, MKN-45 and HGC-27) compared with one normal gastric mucosa cell line, GES. The expression of miR-329 was further examined in 40 paired GC and adjacent non-tumor gastric tissues through qRT-PCR. The expression of miR-329 in GC tissues was significant lower than in adjacent tissues (Figure 1B, *p* < 0.001). The decrease of miR-329 was found in 34 of 40 compared with the corresponding non-tumor tissues (Figure 1C). Moreover, the level of miR-329 was significantly lower in GC patients with late stage disease (Figure 1D).

**Figure 1:** miR-329 was down-regulated in GC **(A)** qRT-PCR analysis of the expression of miR-329 in four cell lines (MGC-803, SGC-7901, MKN-45 and HGC-27) and one normal gastric mucosa cell line (GES). **(B)** Expression of miR-329 in GC tissues was lower than that in non-tumor adjacent tissues. **(C)** miR-329 was detected in 40 GC patients by real-time PCR. Data are presented as log 2 of fold change of GC tissues relative to non-tumor adjacent tissues. **(D)** The Statistical analysis of the association between miR-329 level and pTNM stage (I, II, III and IV). The endogenous U6 snRNA was used as an internal control. *p < 0.05, and **p < 0.01, ***p < 0.001.

### Exogenetic overexpression of miR-329 suppressed GC cell growth

Increased expression of miR-329 upon transfection in the GC cell lines (HGC-27 and MGC-803) was confirmed by qRT-PCR (Figure 2A and 2B). We discovered that miR-329-transfected cells had much fewer growth percentages than that in the scramble mimics-transfected cells; conversely, miR-329 inhibitor significantly accelerated the cell proliferation of MGC-803 and HGC-27 (Figure 2C and 2D).

The article "By downregulating TIAM1 expression, microRNA-329 suppresses gastric cancer invasion and growth" was retracted in 2026. Reasons: plagiarized images; duplicated images; overlap with other authors' work; unreliable results or conclusions.

**Figure 2:** Exogenetic overexpression of miR-329 suppressed GC cell growth **(A)** Expression levels of miR-329 in the MGC-803 cells were examined by qRT-PCR after transfection of 20 nmol/l miR-329 mimics, or scramble or control or inhibitors. **(B)** Expression levels of miR-329 in the HGC-27 cells were examined by qRT-PCR after transfection of 20 nmol/l miR-329 mimics, or scramble or control or inhibitors. **(C)** Growth of MGC-803 cells shown after transfection with 20 nmol/l miR-329 mimics, miR-329 inhibitor, or scramble or control. Growth index was assessed at 0, 1, 2 and 3 days. **(D)** Growth of HGC-27 cells shown after transfection with 20 nmol/l miR-329 mimics, miR-329 inhibitor, or scramble or control. Growth index was assessed at 0, 1, 2 and 3 days. *p < 0.05, and **p < 0.01, ***p < 0.001.

### Overexpression of miR-329 inhibited GC cell migration and invasion

Migration assay analysis has shown that overexpression of miR-329 can enhance both the HGC-27 and MGC-803 cells migration; miR-329 inhibitor significantly accelerated the cell migration of MGC-803 and HGC-27 (Figure 3A and 3B). Invasion assay was then performed to evaluate the effect of miR-329 on the cell invasiveness in miR-329 overexpressing HGC-27 and MGC-803 cells and showed attenuated invasiveness of GC cells; whereas miR-329 inhibitor increased cell invasion (Figure 3C and 3D).

**Figure 3:** Overexpression of miR-329 inhibited GC cell migration and invasion **(A)** MGC-803 cells were transfected with 20 nmol/l miR-329 mimics, miR-329 inhibitor, or scramble or control for 24 h, and migration assay was performed. Relative ratio of migrate cells per field is shown. **(B)** miR-329 inhibited the migration of GC HGC-27 cells; Relative ratio of migrate cells per field is shown. **(C)** MGC-803 cells were transfected with 20 nmol/l miR-329 mimics, miR-329 inhibitor, or scramble or control for 24 h, and invasion assay was performed. Relative ratio of invasive cells per field is shown. **(D)** miR-329 inhibited the invasion of GC HGC-27 cells; Relative ratio of migrate cells per field is shown. *p < 0.05, and **p < 0.01, ***p < 0.001.

### miR-329 targets TIAM1 in GC cells

The 3′UTR of TIAM1 messenger RNA contains a complementary site for the seed region of miR-329 (Figure 4A). The effect of miR-329 on the translation of Tiam1 mRNA into protein was assessed by luciferase reporter assay in HGC-27 cells (Figure 4B). As shown in Figure 3C, miR-329 mimics could significantly decrease TIAM1 mRNA expression; conversely, miR-329 inhibitor significantly accelerated the TIAM1 mRNA expression (Figure 4C). The protein level of TIAM1 was substantially decreased after ectopic overexpression of miR-329 in HGC-27 cell line as evidenced by western blot assays (Figure 4D). On the other hand, knocking down of miR-329 by miR-329 inhibitor in HGC-27 cells increased protein levels of TIAM1 (Figure 4D).

The article "By downregulating TIAM1 expression, microRNA-329 suppresses gastric cancer invasion and growth" was retracted in 2026. Reasons: plagiarized images; duplicated images; overlap with other authors' work; unreliable results or conclusions.

**Figure 4:** miR-329 targets TIAM1 in GC cells **(A)** The 3′UTR of TIAM1 mRNA contains the binding sequences of miR-329. **(B)** Relative luciferase activity of the indicated TIAM1 reporter construct in HGC-27 cells is shown. Firefly luciferase values were normalized to Renilla luciferase activity and plotted as relative luciferase activity. **(C)** Overexpression of miR-329 significantly reduced the TIAM1 mRNA levels in the HGC-27 cells and miR-329 inhibitor significantly promoted the TIAM1 mRNA levels in the HGC-27 cells using qRT-PCR. **(D)** Western blot was performed to examine the effects of miR-329 mimics or inhibitors on the expression of TIAM1. GAPDH was also detected as a loading control. ***p < 0.001.

### miR-329 regulated cell proliferation and invasion through inhibiting TIAM1

The TIAM1 expression vector pcDNA3-TIAM1 was used to restore TIAM1 expression. The protein level of TIAM1 was reduced when miR-329 mimics were transfected with pcDNA3-TIAM1 after 48 h in both HGC-27 and MGC-83 cells (Figure 5A). As expected, the ectopic expression of TIAM1 rescued the miR-329-mediated inhibition of cell proliferation and migration in HGC-27 and MGC-83 cells (Figure 5B, 5C and 5D).

**Figure 5:** miR-329 regulated cell proliferation and invasion through inhibiting TIAM1 **(A)** miR-329 decreased TIAM1 protein levels in both the MGC-803 and HGC-27 cells. **(B)** Cell proliferation was determined by CCK-8 assay. The ectopic expression of TIAM1 rescued the miR-329-mediated inhibition of cell proliferation in HGC-27 cells. **(C)** The ectopic expression of TIAM1 rescued the miR-329-mediated inhibition of cell proliferation in MGC-803 cells. **(D)** The over-expression of TIAM1 rescued the miR-329-mediated inhibition of cell invasion in both the HGC-27 and MGC-803 cells. *p < 0.05, and **p < 0.01, ***p < 0.001.

### TIAM1 was inversely expressed with miR-329 in GC patients

As shown in Figure 6A, the mRNA expression of TIAM1 was significantly up-regulated in four cell lines (MGC-803, SGC-7901, MKN-45 and HGC-27) compared with one normal gastric mucosa cell line, GES. The protein expression of TIAM1 was also up-regulated in four cell lines (MGC-803, SGC-7901, MKN-45 and HGC-27) compared with one normal gastric mucosa cell line, GES (Figure 6B). The protein level of TIAM1 was analyzed in four miR-329 downregulated GC tissues. The levels of these proteins were evidently upregulated in GC as compared with the matching non-neoplastic tissues (Figure 6C). To further validate our findings, the levels of TIAM1 were measured in 20 of human primary GC and pair-matched peritumoral gastric tissues. Comparison of miR-329 levels and levels corresponding to TIAM1 in GC exhibited significantly inverse correlation between TIAM1 and miR-329 (*r*2 = 0.329, *P* = 0.0081) (Figure 6D).

The article "By downregulating TIAM1 expression, microRNA-329 suppresses gastric cancer invasion and growth" was retracted in 2026. Reasons: plagiarized images; duplicated images; overlap with other authors' work; unreliable results or conclusions.

**Figure 6:** TIAM1 was inversely expressed with miR-329 in GC patients **(A)** qRT-PCR analysis of the mRNA expression of TIAM1 in four cell lines (MGC-803, SGC-7901, MKN-45 and HGC-27) and one normal gastric mucosa cell line (GES). **(B)** The protein level of TIAM1 in four cell lines (MGC-803, SGC-7901, MKN-45 and HGC-27) and one normal gastric mucosa cell line (GES) was tested using western blot. **(C)** Western blot analysis of TIAM1 protein expression in four patients whose miR-329 expression was downregulated in GC tissues (C) compared to corresponding adjacent nonneoplastic tissues (N). **(D)** Inverse correlation between TIAM1 level and miR-329 expression in 20 GC samples.

### miR-329 inhibited the growth of HGC-27-engrafted tumors

To investigate the therapeutic effect of miR-329 on gastric tumorigenicity *in vivo*, ~3 × 10^6^ HGC-27 cells were inoculated subcutaneously in posterior flanks of immunocompromised “nude” mice. When tumors reached 50 mm^3^, synthetic miR-329 or scrambled oligonucleotides were injected directly into the tumors. The tumors were injected every 3 days for a total of five times. After 4 weeks, we found that injection with miR-329 inhibited the growth of HGC-27-engrafted tumors with respect to scrambled oligonucleotides-treated tumors (Figure 7A). In agreement with the tumor growth curve, the volumes and weights of tumors treated by miR-329 mimics were significantly lower than scrambled mimics-injected tumors (Figure 7B and 7C). We also performed western blot to detect the protein expression of TIAM1 in randomly selected xenograft mouse tumors and found that miR-329 mimics-injecting tumors expressed lower levels of TIAM1 than scramble controls (Figure 7D).

**Figure 7:** miR-329 inhibited the growth of HGC-27-engrafted tumors **(A)** Representative tumors were photographed at 15 days after the first treatment with miR-329 mimic or sramble. Scale bar: 5 mm. **(B)** Tumor weight averages between scrambled and miR-329 mimics-treated mice groups at the end of the experiment (day 25), Five mice in each group. **(C)** Graph representing tumor volumes at the indicated days during the experiment for the two groups: scrambled mimics, miR-329 mimics. **(D)** Injection of miR-329 reduced TIAM1 protein levels in HGC-27 xenograft tumors. Represented are 2 tumors from each group. *p < 0.05, and **p < 0.01, ***p < 0.001.

The article "By downregulating TIAM1 expression, microRNA-329 suppresses gastric cancer invasion and growth" was retracted in 2026. Reasons: plagiarized images; duplicated images; overlap with other authors' work; unreliable results or conclusions.

## DISCUSSION

Tumor invasion and metastasis is a complex and multistep process [24, 25]. More and more researches have documented that miRNAs serve as master regulators of gene expression in a sequence-specific fashion and have essential roles in multiple biological processes, including cell differentiation, proliferation, angiogenesis, invasion and migration [26–30]. Those miRNAs that are overexpressed in tumors may be oncogenes, and generally participate in tumor suppressor genes underexpressed [31–33]. Although oncogenic and tumor suppressive roles of several miRNAs have been characterized in several different types of tumors, the exact molecular mechanism by which miRNAs modulate the process of tumorigenesis is not yet fully elucidated. In this study we demonstrate that miR-329 was frequently downregulated in human GC cancer, and that miR-329 was significantly associated with late stage. Further studies showed that overexpression of miR-329 suppressed GC cell proliferation, migration, and invasion in GC cells MGC-803 and HGC-27. As for the mechanism, our results indicated that miR-329 directly targeted TIAM1 to inhibit cell invasiveness in GC cells. Moreover, our investigation for the expression of TIAM1 and miR-329 in 20 GC patients indicated that there was an inverse correlation between miR-329 and TIAM1 levels. Importantly, overexpressing miR-329 ameliorated progression of GC in an established experimental xenograft model. These findings suggest that miR-329 has an important role in inhibiting the development and progression of GC.

Recently, several studies reported that the expression of miR-329 was decreased in several different types of cancers, including glioma and neuroblastoma [22, 23]. In glioma, overexpression of miR-329 inhibited cell proliferation of glioma cells by regulating E2F1-mediated inhibition of Akt pathway [23]. Moreover, miR-329 has been found to be a suppressor of angiogenesis by targeting CD146, an endothelial biomarker which was aberrantly upregulated during pathological angiogenesis and acted as a coreceptor of vascular endothelial growth factor receptor 2 (VEGFR2) to promote disease progression [34]. Furthermore, miR-329 was decreased in metastatic neuroblastoma tumor tissues compared with matched primary tumor tissues. Forced overexpression of miR-329 substantially suppressed cell proliferation, colony formation, migration, and invasion of neuroblastoma cells by regulating Lysine-specific demethylase 1 (KDM1A) [22]. In the other study, increased miR-329 was observed in oral squamous cell carcinoma specimens compared to the matched tissue ulcerative colitis, suggesting its function as an oncogene [35]. Our data demonstrated that the downregulation of miR-329 frequently exists in GC tissue and cell lines, suggesting a tumor suppressive role of miR-329 in GC development. To further verify the role of miR-329 in the development of GC, cell transfection was performed. Upregulation of miR-329 significantly inhibited cell proliferation, migration, and invasion in GC cell lines, indicating that repression of miR-329 might promote tumor progression in gastric carcinogenesis.

The article "By downregulating TIAM1 expression, microRNA-329 suppresses gastric cancer invasion and growth" was retracted in 2026. Reasons: plagiarized images; duplicated images; overlap with other authors' work; unreliable results or conclusions.

To explore the molecular mechanism underlying miR-329 function, it is important to identify its target gene. Recently, several novel targets of miR-329 have been confirmed including E2F1, CD146 and KDM1A [22, 23, 34]. In our study, TIAM1 was identified as a target gene of miR-329 in GC. We here performed *in vitro* and *in vivo* studies to demonstrate that miR-329 can regulate GC cell proliferation and invasion through targeting TIAM1. TIAM1 has been implicated as a ubiquitous Rac activator that participates in several cellular processes in normal physiological processes as well as in disease processes, such as invasion and metastasis of tumor cells [36, 37]. Tiam1 activation can promote cell proliferation, migration, invasion, and metastasis in a variety of cancers, such as breast cancer, prostate cancer, hepatocellular carcinoma, colon carcinoma, and renal carcinoma [38–43]. Previous study has shown that the expression of TIAM1 is upregulated in GC compared with adjacent pair-matched non-tumor tissues, and postoperative survival analysis indicated that patients with strong TIAM1 expression had lower disease-specific survival rates than those with negative TIAM1 expression [38, 44]. The dual-luciferase reporter assays indicated that TIAM1 was one of the functional downstream targets of miR-329, which suggested that miR-329 suppressed TIAM1 expression by interacting with the 3′UTR of TIAM1 mRNA. Moreover, ectopic expression of TIAM1 significantly increased the proliferation and invasion of HGC-27 and MGC-803 cells overexpressing miR-329. These results demonstrate that TIAM1 is a functional target gene of miR-329 in GC.

We have also analyzed the correlation between miR-329 expression and the expression of TIAM1 in 20 primary GC samples. Consistent with the cell line data, TIAM1 were enriched in the primary GC tissues that inversely correlated to miR-329 levels. However, further studies using large numbers of primary GC samples will be needed to confirm this interaction.

There are no study has tested whether miR-329 could reduce tumorigenicity in a xenograft model, we tested the tumor-suppressive role of miR-329 *in vivo* through direct miRNA mimics injection and found that miR-329 significantly inhibited the growth of GC cells. Further western blot analysis in xenograft carcinoma tissues demonstrated the negative regulation of miR-329 to TIAM1 suggesting that miR-329 might be better therapeutic choices in GC.

The article "By downregulating TIAM1 expression, microRNA-329 suppresses gastric cancer invasion and growth" was retracted in 2026. Reasons: plagiarized images; duplicated images; overlap with other authors' work; unreliable results or conclusions.

In conclusion, the identification of miR-329 as a tumor suppressive miRNA in human GC that acts by repressing TIAM1 provides additional evidence of a pivotal role for miRNAs in GC tumorigenesis and progression. Given that miR-329 is downregulated in GC, the introduction of this mature miRNA into the tumor tissue could serve as a therapeutic strategy by reducing the expression of target genes. MiRNA-based therapeutic patterns are still in their infancy; however, our findings are encouraging and suggest that this miRNA could be targeted for the development of a treatment for patients with GC in the future.

## MATERIALS AND METHODS

### Patients and samples

This study was approved by the Clinical Research Ethics Committee of the Peking Union Medical College Hospital. Each subject was signed with informed consent. No patients had received chemotherapy or radiotherapy before surgery. The tissue samples for all experiments were approved to be used by all the patients and by the Ethics Committee of the institution. Gastric cancer tissues and their morphologically normal tissues (located > 3 cm from the tumor) were collected from 40 GC patients undergoing surgery at the Cancer Hospital of the Chinese Academy of Medical Sciences between 2013 and 2014. Tissue samples collected were divided into two parts. One part immediately stored in liquid nitrogen until RNA or protein extraction, and the other part was fixed in 10% formalin for the histopathological diagnosis. The characteristics of the patients are described in Table S1.

### Cell lines and cell culture

The human GC cell lines (MGC-803, SGC-7901, MKN-45 and HGC-27) and one normal gastric mucosa cell line (GES) were purchased from the American Type Culture Collection (ATCC, Manassas, VA, USA). Four of the cell lines (SGC-7901, MKN-45, HGC-27 and GES) were cultured in Roswell Park Memorial Institute (RPMI)-1640 (PAA) containing 10% v/v fetal bovine serum (FBS; Trace Scientific, Melbourne, Australia), the other cell line MGC-803 in Dulbecco's modified Eagle medium (Gibco; Invitrogen; Life Technologies, Germany) containing 10% FBS. All the cell lines were incubated at 37°C in a humidified atmosphere with 5% carbon dioxide.

### RNA extraction and quantitative real-time PCR

Total RNA was extracted by Trizol reagent (Invitrogen, Carlsbad, CA) according to the manufacturer's protocol. Quantitative real-time PCR (q-PCR) was performed by Taqman probes (Invitrogen) in the Bio-Rad IQ5 real-time PCR system according to the manufacturer's instructions in order to measure the level of miR-329. The 2^−ΔΔCT^ method was used in the analysis of PCR data. The endogenous U6 snRNA was used as an internal control. The primers were described in Table S2.

The article "By downregulating TIAM1 expression, microRNA-329 suppresses gastric cancer invasion and growth" was retracted in 2026. Reasons: plagiarized images; duplicated images; overlap with other authors' work; unreliable results or conclusions.

### Oligonucleotides and transfection

MiR-329 mimics/inhibitors and negative control molecules (scramble control mimic and inhibitor) were purchased from Dharmacon (Austin, TX). Cell transfection was performed with DharmFECT1 (Dharmacon) at a final concentration of 20 nM. Medium was changed after 6 h. After being cultured for 48 h, cells were harvested for Western blot and qRT-PCR analyses.

### Cell proliferation assay

Cells were cultured in 10% CCK-8 (DOJINDO) diluted in normal culture media at 37°C until visual color conversion appeared. Quantification was carried out on a microtiter plate reader (Spectra Rainbow; Tecan) according to the manufacturer's instructions. Cell proliferation rates were calculated at 0, 24, 48 and 72 h posttransfection.

### Cell migration and invasion assay

HGC-27 and MGC-803 cells were grown to 50–70% confluence. For the migration assays, cells were transfected with miR-329 mimics or control mimics, inhibitor or control and then added into the upper chamber of the insert (BD Bioscience, 8-μm pore size). For the invasion assays, cells were added into the upper chamber of the insert precoated with Matrigel (BD Bioscience). Cells were incubated in medium without serum, and in medium with 10% FBS served as chemo attractant in the lower chamber in both assays. After several hours of incubation, cells that did not migrate or invade through the pores were carefully wiped out with cotton wool. After being stained by 20% methanol and 0.2% crystal violet, the inserts were imaged and counted.

### Western blot

After being separated on 12% SDS-PAGE gel, proteins were transferred onto a nitrocellulose membrane (Bio-Rad, Hercules, USA). After being blocked with 5% non-fat milk, the membrane was incubated with anti-TIAM1 antibody or anti-GAPDH (Santa Cruz, CA). The membrane was then washed extensively and incubated with a goat anti-mouse secondary antibody (Pierce, IL, USA). The proteins were detected with ECL reagents (Pierce).

### Luciferase reporter assays

By cloning human TIAM1 mRNA sequence into pMIR-Report construct (Ambion, Austin, USA), luciferase reporter construct was made. Wild type or mutant TIAM1 mRNA fragment (from 26 to 32) was amplified and cloned into the luciferase reporter via SpeI and HindIII sites. Using the JetPRIME reagent (Polyplus-transfection), HGC-27 cells were co-transfected with 20 nM single-stranded miRNA mimics or negative control oligonucleotides, 20 ng of firefly luciferase reporter and 10 ng of pRL-TK (Promega, USA). Cells were collected after being transfected for 24 hours and analyzed using Dual-Luciferase Reporter Assay System (Promega).

The article "By downregulating TIAM1 expression, microRNA-329 suppresses gastric cancer invasion and growth" was retracted in 2026. Reasons: plagiarized images; duplicated images; overlap with other authors' work; unreliable results or conclusions.

### *In vivo* studies

Animal xenograft model studies were performed according to institutional guidelines; 3 × 10^6^ HGC-27 viable cells were injected subcutaneously into the posterior flanks of 6-week female nude mice, five mice per group. When tumor size reached 50 mm^3^, miRNA mimics (miR-329 or scrambled control) diluted in Lipofectamine 2000 (Invitrogen) solution (100 nmol mimics in 100 μl total volume) were directly injected into the tumors, respectively. These tumors were injected every 3 days for a total of six times. Tumor diameters were measured after 10 days of injection and then measured every 3 days. On the 25^th^ days after injection, mice were killed. Tumors were collected and weighted after necropsy. Tumor volume was calculated as follows: length × width 2 × 1/2.

### Statistics

The statistical analysis of miR-329 expression between GC tissues and control tissues was evaluated by independent sample *t*-test (two tailed). Correlation of miR-329 expression with patients' clinicopathological variables was evaluated by independent sample *t*-test (two tailed) or one-way analysis of variance, followed by Tukey post hoc test. All the analyses were completed using software SPSS17.0. *P* ≤ 0.05 was considered as statistically significant.

## SUPPLEMENTARY TABLES


